The article "Curcumin improves age-related and surgically induced osteoarthritis by promoting autophagy in mice" was retracted in 2022. Reason: duplicated images.

# Curcumin improves age-related and surgically induced osteoarthritis by promoting autophagy in mice

**DOI:** 10.1042/BSR20171691

**Published:** 2018-07-03

**Authors:** Guowang Zhang, Jiaqing Cao, Erzhu Yang, Bo Liang, Jianing Ding, Jiaming Liang, Jianguang Xu

**Affiliations:** Department of Orthopedic Surgery, Shanghai Jiao Tong University Affiliated Sixth People’s Hospital, Shanghai 200233, China

**Keywords:** autophagy, curcumin, Osteoarthritis

## Abstract

Reduced autophagy has been implied in chondrocyte death and osteoarthritis. Curcumin (Cur) owns therapeutic effect against osteoarthritis (OA) and enhances autophagy in various tumor cells. Whether the cartilage protection of curcumin is associated with autophagy promotion and the potential signaling pathway involved remains unclear. The present study aimed to investigate the role of autophagy in the anti-OA activity of curcumin using spontaneous and surgically induced OA mice model. Spontaneous and surgically induced OA mice model was established and treated with Cur. Articular cartilage destruction and proteoglycan loss were scored through Safranin O/Fast green staining. Apoptotic cell death was detected with TUNEL (terminal deoxynucleotidyl transferase-mediated dTUP-biotin nick end labeling assay) staining and Western blot for caspase-3, Bcl-2 associated X protein (Bax), and Bcl-2 (B-cell lymphoma-2). Light chain 3 (LC3) immunohistochemistry was used to evaluate autophagy. *In vitro*, primary chondrocytes were treated with interleukin 1 beta (IL-1β) and Cur. Autophagy was inhibited using 3-methyladenine. Apoptosis and autophagy were detected using flow cytometry and Western blotting assay. Curcumin treatment enhanced autophagy, reduced apoptosis, and cartilage loss in both OA models. *In vitro*, curcumin treatment improved IL-1β induced autophagy inhibition, cell viability decrease, and apoptosis. Mechanistically, *in vivo* studies suggested curcumin promoted autophagy through regulating Akt/mTOR pathway. In conclusion, our results demonstrate that curcumin-induced autophagy via Akt/mTOR signaling pathway contributes to the anti-OA effect of curcumin.

## Introduction

Osteoarthritis (OA) is a degenerative and progressive disease with substantial pain and disability in worldwide. Prevalence was higher in females than males. Life lived with disability (YLDs) for hip and knee OA increased from 10.5 million in 1990 to 17.1 million in 2010 [1]. It is characterized by inflammation of synovial membrane, modification of the subchondral bone structure, degradation of articular cartilage which is often reflected by loss of cartilage extracellular matrix, and reduced cartilage cellularity [2,3]. Despite the great attempts made on reducing the prevalence of OA, there is no effective treatment or cure that reverses disease progression [4]. Plus, a majority of currently used drugs for OA has serious side effects, especially with long-term use. Novel and safe treatment for OA are thus in high demand and are subject of the present study.

The article "Curcumin improves age-related and surgically induced osteoarthritis by promoting autophagy in mice" was retracted in 2022. Reason: duplicated images.

Curcumin is an active component extracted from dried rhizomes of *Curcuma longa*. Since curcumin owns anti-inflammatory and antioxidative properties, it has been widely used in Traditional Chinese Medicine for ameliorating OA [5]. Curcumin has been reported to be potential inhibitor of NF-κB and JNK signaling pathways, and activators of STAT in human and bovine primary chondrocytes [6–8]. It has recently been reported that curcumin regulates activation of AMPK signaling pathway in aging-related vascular dysfunction in old mice [9]. In addition, curcumin can suppress the expression of genes related to matrix metalloproteinases (MMPs) that play critical role in disruption of cartilage extracellular matrix [10–12].

With removing the intracellular unfolded proteins and damaged organelles, autophagy plays crucial role in cellular self-protection [13–15]. However, autophagy owns both beneficial and pathogenic effects in cell mechanism and homeostasis [16]. Importance of autophagy and its functional mechanism was well established in relation to cardiovascular disease [17], pancreatic abnormality [18], neurodegenerative disease [19], liver cancer [20], and aging and aging-related disease [21]. Along with chondrocyte aging and senescence, autophagy plays potential role in the development and progression of OA [22]. Recent study demonstrated that curcumin suppresses chondrocyte apoptosis through activation ERK1/2-induced autophagy *in vitro* [23]. However, to best of our knowledge, no study ever reported the protective effect of autophagy, which is induced by curcumin, in OA animals or patients. Thus, in the present study, we attempt to evaluate the therapeutic effect of curcumin in two different OA mice models by elucidating its impact on autophagy.

## Materials and methods

### Animal model and treatment

All animal experiments were conducted in accordance with the approval of the Institutional Animal Care and Use Committee at Shanghai Jiao Tong University Affiliated Sixth People’s Hospital. A total number of 50 C57BL/6 male mice were recruited into the present study (*n*=10). For the aging-related OA mice model, C57BL/6 male mice were given tamoxifen at a dose of 1 mg/10 g body weight for 5 days [24] at age of 8 weeks and kept under normal circumstances up to 12 months of age (*n*=10; aging control group). Mice were given dietary curcumin (0.5%) for 12 months (*n*=10; aging curcumin group) [25]. For the surgery-induced OA model, 10-week-old mice were subjected to destabilization of the medial meniscus (DMM) in right knee joints and mice were given corn oil only (*n*=10; surgical vehicle control group). In sham operational group, the medial meniscus of mice was visualized but not dissected (*n*=10; sham control group). Immediately after the surgery, mice were subjected to oral administration of 50 mg/kg curcumin (Sigma) dissolved in corn oil administered via oral gavage, once daily for 8 weeks (*n*=10; surgical curcumin group) [26]. There were ten mice in each group and all animals were kept in 12-h day/12-h night cycle with free access to food and water.

The article "Curcumin improves age-related and surgically induced osteoarthritis by promoting autophagy in mice" was retracted in 2022. Reason: duplicated images.

### Terminal deoxynucleotidyl transferase-mediated dTUP-biotin nick end labeling assay (TUNEL) staining

For *in situ* apoptosis examination, animals were killed at 8 weeks after curcumin treatment. The knee joint samples were fixed in formalin, decalcified, and embedded in paraffin. Serial 4-μm sections were cut across the medial femorotibial joint and mounted. After being dewaxed in xylene and dehydrated with graded concentrations of alcohols, sections were subjected to chondrocyte apoptosis analysis with TUNEL staining using *in situ* Apoptosis Detection Kit (CHEMICON, CA, U.S.A.) in accordance with the manufacturer’s instructions. The signals of positive staining were detected by light microscopy. TUNEL staining (in green) and DAPI nuclear counterstaining (in blue) were performed to assess chondrocyte apoptosis. The apoptotic ratio (%) was measured: it is defined as ratio between the total number of positive nuclei and the total number of the present cells in one plane in each section. We selected three sections (*n*=3) from each specimens. The average apoptotic ratio (%) for the different groups was then compared and statistically analyzed.

### Histological examination and immunohistochemistry

Cartilage degeneration induced by aging or surgery was assessed using Safranin O/Fast green staining. Samples were cut through the medial knee joints and 5-μm sections (*n*=5) were used. Sections were stained with Safranin O visualized under light microscope. Proteoglycan depletion in cartilage and subchondral plate thickness was assessed in accordance with the Mankin’s scoring methods with slight modification (on a scale of 0–3, but total score 13 did not change).

Knee joint sections were deparaffinized using conventional method and endogenous peroxidase activity was blocked with 3% H_2_O_2_. Sections were incubated with rabbit anti-LC-3 polyclonal antibody (1:500; Abcam, Hangzhou, China) followed by incubation with corresponding secondary antibody (Abcam, Hangzhou, China) and stained with DAB kit (Sangon Biotech, Shanghai, China).

The article "Curcumin improves age-related and surgically induced osteoarthritis by promoting autophagy in mice" was retracted in 2022. Reason: duplicated images.

### Chondrocyte isolation and treatment

The primary chondrocytes were isolated from dissected knee joint of normal mice using 0.1% collagenase (Gibco) as described elsewhere [27]. Chondrocytes were maintained in DMEM supplemented with 10% fetal bovine serum. For *in vitro* experiments, serum starved primary isolated chondrocytes were either treated with 10 ng/ml IL-1β for 24 h or pretreated with 10 μM curcumin for 4 h and co-treated with 10 ng/ml IL-1β and 10 μM curcumin for the same time periods [28]. To inhibit autophagy, the chondrocytes were pretreated with 3-methyladenine (3-MA; 10 nM, Sigma–Aldrich, MO, U.S.A.) for 2 h before treatment with curcumin or IL-1β. Three independent experiments were performed in triplicate.

### CCK-8 assay

Cell viability was determined by cell-counting kit-8 (CCK-8) assay (Dojindo, Japan). Briefly, after treatment cells were seeded on to 96-well plates with the density of 7000/well and incubated for 24 h. CCK-8 solution was added into each well and incubated for 1 h at 37°C at dark place. The OD values were read at dual wavelengths of 450 and 630 nm to determine cell viability using a microplate reader (Thermo Fisher Labsystems). Three independent experiments were performed in triplicate.

### Annexin V/PI staining and flow cytometry

For *in vitro* apoptotic analysis, Annexin V/PI dual staining assay was performed. After treatment, cells were harvested and incubated with 2 μg/ml of Annexin-FITC and 2.5 μg/ml of PI (Santa Cruz Biotechnology, CA, U.S.A.) according to manufacturer’s instructions. Cells were analyzed using FACS Calibur (BD Biosciences). Three independent experiments were performed in triplicate.

### Quantitative RT-PCR

Total mRNAs were extracted from chondrocytes using TRIzol (Invitrogen, CA, U.S.A.). RNA quality and concentration were determined using NanoDrop 2000 (Thermo Fisher Scientific). Five hundred nanograms of total mRNA was used to synthesize cDNA in total volume of 20 μl of reaction solution using cDNA-synthesis kit (Bio-Rad Laboratories, CA, U.S.A.). Real-time PCR was performed using SYBR green PCR Master Mix (Takara, Dalian, China) in triplicate. The amplification was conducted in accordance with the following cycling conditions: 95°C for 5 min, 40 cycles of denaturation, at 95°C for 20 s and annealing and extension at 72°C for 20 s. The gene expression was calculating in accordance with the 2^−ΔΔ*C*^_t_ methods. The results were analyzed after target gene expression was normalized to β-actin expression. Three independent experiments were performed in triplicate.

### Western blot analysis

Cytosolic proteins were extracted from mouse chondrocytes using RIPA lysis buffer containing a protease inhibitor cocktail. Equal amount of proteins were separated on SDS-PAGE gels and subjected to electrophoresis. The proteins were transferred onto polyvinylidene difluoride membranes and blocked with 5% nonfat milk at room temperature for 4 h. Membranes were incubated with appropriate primary antibodies for overnight. After being washed with TBST, membranes were incubated with HRP-conjugated secondary antibodies at room temperature for 2 h. At the end, membranes were washed with TBST and chemiluminescent signal was detected using a Gel Doc 2000 Imager (Bio-Rad, U.S.A.). All primary and secondary antibodies were purchased from Abcam (Abcam, Hangzhou, China).

The article "Curcumin improves age-related and surgically induced osteoarthritis by promoting autophagy in mice" was retracted in 2022. Reason: duplicated images.

### Statistical analysis

All statistical analysis were conducted using SPSS package version 17.0. The data were presented as mean ± SD. Significant differences in mean values between two groups were assessed by Student’s *t* test. Comparisons among multiple groups were made using analysis of variance (ANOVA) test. For both Western blot and TUNEL staining analysis, we performed one-way ANOVA test to compare the difference. Two-sided *P* values < 0.05 were considered statistically significant.

## Results

### Curcumin retards aging-related cartilage degradation in mouse articular cartilage

Articular cartilage from age-related OA mice exhibited homogeneous Safranin O staining in all zones. At age of 12 months, mice developed OA-like phenotypes, such as disrupted subchondral bone structure and low cell density (Figure 1A). The mice with curcumin treatment, however, showed the significant increase in Safranin O staining and increase in cartilage thickness compared with mice in nontreatment group (*P*<0.05) (Figure 1B,C).

**Figure 1:** Curcumin reduced the cartilage degradation in spontaneous aging-related OA mice (**A**) Safranin O staining of articular cartilage obtained from C57BL/6 male mice kept in normal condition for 12 months with (*n*=10) and without (*n*=10) curcumin treatment. (**B**) Relative cartilage thickness and (**C**) Mankin’s score based on staining results. Student’s *t* test was performed to determine the difference between curcumin treatment and control mice; *P<0.05 and **P<0.01 compared with controls.

### Curcumin decreases severity of OA in the knee joints following DMM surgery

We determined the impact of curcumin on DMM-induced OA by evaluating the structural features of articular cartilage with Safranin O staining and Mankin’s score. Four-month-old mice were subjected to DMM surgery-induced OA. Eight weeks after surgery, knee joints of mice in DMM surgery group exhibited OA pathology characterized by reduced Safranin O staining and low cell density (Figure 2A). The mice in the curcumin treatment group showed the amelioration of OA severity as indicated by increased cell density. Based on these observations, we conducted quantitative analysis and found that cartilage thickness was notably lower in DMM group compared with sham controls (*P*<0.05) and curcumin treatment retarded the tissue degradation (*P*<0.05) (Figure 2B). In addition, Mankin’s score was significantly higher in DMM group compared with sham controls (*P*<0.05), and this rise was reduced significantly with curcumin treatment (*P*<0.05) (Figure 2C).

The article "Curcumin improves age-related and surgically induced osteoarthritis by promoting autophagy in mice" was retracted in 2022. Reason: duplicated images.

**Figure 2:** Curcumin reduced the cartilage degradation in DMM surgery-induced OA male mice (**A**) Safranin O staining of articular cartilage obtained from mice after 8 weeks of DMM surgery (*n*=10), sham operation (*n*=10), and curcumin treatment (*n*=10). (**B**) Relative cartilage thickness and (**C**) Mankin’s score based on staining results. One-way ANOVA test was performed to determine difference between sham, DMM, and curcumin treatment mice. **P<0.01 compared with controls; ^##^*P*<0.01 compared with DMM mice.

### Curcumin suppresses chondrocyte apoptosis in knee joints of mice with surgically induced and age-related OA

To further investigate the effect of curcumin on chondrocyte apoptosis in DMM-induced and age-related OA, we conducted TUNEL staining analysis on articular cartilage. Eight weeks after DMM surgery, the OA mice showed the cartilage degradation with notably enhanced chondrocyte apoptosis compared with OA mice in sham control group. TUNEL staining (in green) and DAPI nuclear counterstaining (in blue) were performed to assess chondrocyte apoptosis. With curcumin treatment, mice exhibited the improved cartilage loss with reduced apoptotic cell death as evidenced by reduction in number of TUNEL-positive cells (Figure 3A). Similar trend was observed in spontaneous age-related OA mice, showing less apoptotic cell death with curcumin treatment than mice in nontreated group (Figure 3C). The effect of curcumin on apoptotic activity in OA was further confirmed examining apoptosis-related markers by Western blot. In both OA model, surgically induced and age-related, activation of caspase-3 as well as Bax/Bcl2 ratio was suppressed with curcumin treatment (*P*<0.05) (Figure 3B,D).

**Figure 3:** Curcumin inhibits apoptotic chondrocyte death in age-related and surgically induced OA mice TUNEL staining of articular cartilage explants in (**A**) surgically induced (*n*=10) and (**C**) aging-related OA mice (*n*=10). (**B** and **D**) Relative protein expression of cleaved caspase-3 and Bax/Bcl-2 of articular cartilage tissues obtained from surgically induced and aging-related OA mice examined by Western blot analysis. One-way ANOVA test was performed to determine difference between sham, DMM, and curcumin treatment groups; **P<0.01 compared with sham or normal control and ^##^*P*<0.01 compared with DMM.

The article "Curcumin improves age-related and surgically induced osteoarthritis by promoting autophagy in mice" was retracted in 2022. Reason: duplicated images.

### Curcumin enhances chondrocyte autophagy in knee joints of mice with surgically induced and age-related OA

Autophagy is another protective mechanism in normal cartilage. To investigate the effect of curcumin on autophagy, we carried out immunohistochemistry analysis on LC-3 expression in joint tissues from both type of OA mice, spontaneous (Figure 4B) and surgically induced model (Figure 4A). The mice in curcumin treatment group displayed an obvious increase in LC-3 expression in comparison with mice of DMM-induced OA group and aging-related OA group with no treatment. This observation was further confirmed by examining the expression level of autophagy-related markers, LC-I/II, and Beclin1, using Western blot analysis. In both OA models, the expression of LC-I/II and Beclin1 was significantly increased, while the expression of p62 was significantly reduced with curcumin treatment compared with mice without treatment (*P*<0.05) (Figure 4C,D).

**Figure 4:** Curcumin effectively promotes chondrocyte autophagy in aging-related and surgically induced OA mice Immunohistochemical staining of LC3 protein of articular cartilage tissue obtained from (**A**) surgically induced (*n*=10) and (**B**) aging-related OA mice (*n*=10). (**C** and **D**) Western blot analysis of LC3 and Beclin 1 protein expression level in articular cartilage tissue obtained from surgically induced and aging-related OA mice. One-way ANOVA test was performed to determine difference between sham, DMM, and curcumin treatment groups; *P<0.05 and **P<0.01 compared with sham or normal control; ^##^*P*<0.01 and ^#^*P*<0.05 compared with DMM.

### Curcumin modulates autophagy in chondrocytes via AKT/mTOR pathway

The expression level of mTOR, Akt, and p-P70S6k was higher in surgically induced and spontaneous OA mice, and expression level of that was significantly reduced with curcumin treatment compared with nontreated mice (*P*<0.05) (Figure 5A,B). The phosphorylation sites analyzed for Akt and mTOR are Ser473 and Ser 2448 respectively [29]. In order to determine whether regulation of chondrocyte autophagy by curcumin is Akt/mTOR dependent or not, we used nicotine to activate Akt/mTOR signaling pathway. Chondrocytes were pretreated with nicotine (10^−7^ mol/l; Sigma) [30] prior to curcumin treatment. Expression of LC3II was determined with Western blot analysis. As can be seen in Figure 5C, the regulatory effect of curcumin on chondrocyte apoptosis is Akt/mTOR dependent.

The article "Curcumin improves age-related and surgically induced osteoarthritis by promoting autophagy in mice" was retracted in 2022. Reason: duplicated images.

**Figure 5:** Curcumin inhibits Akt/mTOR signaling pathway (**A**) Image of immunoblotting of p-mTOR, p-Akt, and p-P70S6K protein expression in surgically induced (*n*=10) and (**B**) aging-related OA mice (*n*=10) based on Western blot analysis. (**C**) To determine whether regulation of chondrocyte autophagy by curcumin is Akt/mTOR dependent or not, we used nicotine to activate Akt/mTOR signaling pathway by Western blot analysis. One-way ANOVA test was performed to determine difference between sham, DMM, and curcumin treatment groups; **P<0.01 compared with sham or normal control; ^##^*P*<0.01 compared with DMM or nicotine group.

### Autophagy plays an important role in the cartilage protection of curcumin

In order to further validate the potential effect of curcumin on autophagy, we developed *in vitro* OA model using IL-1β in normal primary chondrocytes. The result showed that LC-II/I ratio was significantly lower with IL-1β treatment only compared with controls (*P*<0.05). The expression of LC-II/I was significantly increased with curcumin treatment in IL-1β pretreated chondrocytes (*P*<0.05). LC-II/I ratio was decreased when chondrocytes were pretreated with autophagy inhibitor, 3-MA, compared with curcumin treatment in IL-1β-induced OA chondrocytes (*P*<0.05) (Figure 6A).

**Figure 6:** Curcumin inhibited the IL-1β-stimulated down-regulation of autophagy, IL-1β-stimulated apoptotic chondrocyte death and cartilage matrix degradation (**A**) Relative protein expressions of autophagy-related markers detected by Western blot in primary chondrocytes with different treatments. (**B**) Cell viability detected by CCK-8 assay in differentially treated primary chondrocytes. (**C**) Apoptotic cell proportion examined by flow cytometry in differentially treated primary chondrocytes. (**D**) Relative protein expression of cleaved caspase-3 and Bax/Bcl-2 tested by Western blot. (**E**) Relative mRNA level of MMP13, ADAMTS-5, Col2a1, and Aggrecan examined by quantitative RT-PCR. One-way ANOVA test was performed to determine difference between sham, DMM, and curcumin treatment groups; **P<0.01 compared with normal control; ^##^*P*<0.01 compared with IL-1β treatment group; ^$^*P*<0.05 and ^$$^*P*<0.01 compared with IL-1β+curcumin treatment group.

Cell viability was significantly reduced in cells treated with IL-1β compared with controls (*P*<0.05). Curcumin induced increased cell viability in IL-1β treated cells (*P*<0.05) and the obvious reduction was detected in cells pretreated with 3-MA, compared with ones with curcumin treatment (*P*<0.05) (Figure 6B).

To further investigate the interaction between apoptosis and autophagy, we measured apoptosis level after the autophagy inhibitor treatments. Our results demonstrated that the percentage of apoptotic chondrocytes was significantly increased after IL-1β (*P*<0.05) and reduced with curcumin treatment (*P*<0.05). With treatment of autophagy inhibitor (3-MA), apoptotic rate was significantly increased in IL-1β+curcumin co-treated cells (*P*<0.05) (Figure 6C). To elucidate the antiapoptotic effect of curcumin on OA chondrocytes, we measured apoptosis-related markers. The results showed that expression level of cleaved caspase-3 and Bax/Bcl2 was significantly lower with curcumin treatment in IL-1β-treated cells (*P*<0.05), and when the cells were treated with autophagy inhibitor (3-MA) the apoptotic rate was increased in IL-1β+curcumin co-treated cells (*P*<0.05) (Figure 6D).

In addition, we also determined the mRNA level of genes related to degradation of cartilage matrix in differentially treated chondrocytes using quantitative RT-PCR. Our result demonstrated that mRNA expression of MMP13 and ADAMTS-5 was decreased, while Co12a1 and Aggrecan expression was increased with curcumin treatment in cells co-treated with IL-1β (*P*<0.05). This expression trend was reversed with autophagy inhibitor (3-MA) in IL-1β+curcumin co-treated cells (*P*<0.05) (Figure 6E).

The article "Curcumin improves age-related and surgically induced osteoarthritis by promoting autophagy in mice" was retracted in 2022. Reason: duplicated images.

## Discussion

OA is a slow processing disease with significant articular cartilage loss and fibrillation. Increased age is the major risk factor for the onset and progression of OA [31]. However, ligament rupture in response to joint instability and altered biomechanics resulted in OA 10–15 years later in humans [32,33]. Therefore, surgical instability models have been the most common and popular OA model in laboratory animals [34]. Advantages of surgical models over spontaneous models include a faster onset of disease, decreased variability, and dependence on genetic background [35].

In the present study, we applied both spontaneous and surgically induced OA models in mice in order to eliminate the potential model-bias results and substantial discrepancy in existing models. Our results revealed that curcumin effectively ameliorated the articular cartilage loss in both OA models of mice. Curcumin suppressed apoptosis and enhanced autophagy of chondrocytes in knee joints of both spontaneous and surgically induced OA mice. The enhanced autophagy induced by curcumin is associated with inhibition of Akt/mTOR signaling pathway in both models of OA mice. In order to further validate the impact of curcumin on autophagy, we established OA cell model using inflammatory cytokine and autophagy inhibitor. We found that autophagy plays important role in therapeutic role of curcumin against OA as evidenced by reduced cell viability, increased apoptosis, and degradation of cartilage matrix when autophagy was inhibited.

The article "Curcumin improves age-related and surgically induced osteoarthritis by promoting autophagy in mice" was retracted in 2022. Reason: duplicated images.

The therapeutic effect of curcumin against OA has been well established as evidenced by a great body of clinical experiments [36]. One of the curing mechanisms of curcumin in protection of cartilage loss is that its antiapoptotic role of chondrocyte. A study demonstrated that curcumin inhibits apoptosis in IL-1β-stimulated human chondrocytes *in vitro* examined by immunoblotting and electron microscopy [37]. In the present study, we observed the significantly increased apoptotic chondrocyte in articular cartilage explants *in situ* obtained from spontaneous and surgically induced OA mice.

Aging in mouse and human knee articular cartilage is associated with a reduction in autophagy, as indicated by decreased expression of key regulators of autophagy including ULK1, Beclin 1, and LC3 [38]. Along with aging-related OA, surgically induced OA mice also displayed a reduced autophagy and a related increased apoptosis [39]. Human autophagy gene expression analysis in comparison of healthy and OA cartilage showed the 20 down-regulated autophagy-related genes in OA tissue including LC3 and Beclin1 [40]. These changes were associated with up-regulation of important regulators of cell death/apoptosis [40]. Several literatures have demonstrated that therapeutic role of some bioactive components, such as sucrose [41] and rapamycin [42], in OA was implicated with increased autophagy via regulation of Akt/mTOR signaling pathway. Consistently, our work exhibited that autophagy was reduced, as indicated by down-regulation of LC3 and Beclin1, in both aging-related and surgically induced OA, in which Akt/mTOR was activated. However, these results were revered with curcumin treatment, as evidenced by increased LC3 and Beclin1, as well as the inhibition of Akt/mTOR signaling pathway. In addition, we also conducted *in vitro* experiments designing IL-1β-stimulated OA in primary chondrocyte. The results further validated that the effect of curcumin on autophagy, as indicated by increased autophagy (LC3 and Beclin1), decreased apoptosis (cleaved caspase-3 and Bax/Bcl2), and reduced cartilage matrix degradation (MMP13, ADAMTS-5, Col2a1, and Aggrecan). These results were further confirmed with autophagy inhibitor, showing reversed expression levels of these markers in the presence of 3-MA.

In conclusion, our results demonstrate that curcumin exerts therapeutic role by inducing autophagy via Akt/mTOR signaling pathway in aging-related and surgically induced OA mice.

The article "Curcumin improves age-related and surgically induced osteoarthritis by promoting autophagy in mice" was retracted in 2022. Reason: duplicated images.

## Abbreviations

ANOVA: analysis of variance
Bax: Bcl-2 associated X protein
Bcl-2: B-cell lymphoma-2
CCK-8: cell-counting kit-8
Cur: curcumin
DAPI: 2-(4-amidinophenyl)-6-indolecarbamidine dihydrochloride
DMM: destabilization of the medial meniscus
ECM: extracellular matrix
IL-β: interleukin 1 beta
JNK: c-Jun N-terminal kinase
LC 3: light chain 3
MMP: matrix metalloproteinase
mTOR: mammalian target of rapamycin
NF-κB: nuclear factor kappa B
OA: osteoarthritis
OD: optical density
RIPA: radio immunoprecipitation assay
TBST: Tris buffer solution tween
TUNEL: terminal deoxynucleotidyl transferase-mediated dTUP-biotin nick end labeling assay
